# Follow-Up of High-Grade Glial Tumor; Differentiation of Posttreatment Enhancement and Tumoral Enhancement by DCE-MR Perfusion

**DOI:** 10.1155/2022/6948422

**Published:** 2022-02-01

**Authors:** Tolga Turan Dündar, Ezra Cetinkaya, İsmail Yurtsever, Ömer Uysal, Ayşe Aralaşmak

**Affiliations:** ^1^Bezmialem Vakif University, Department of Neurosurgery, İstanbul, Turkey; ^2^Bezmialem Vakif University, Department of Radiology, İstanbul, Turkey; ^3^Bezmialem Vakif University, Department of Biostatistics and Information, İstanbul, Turkey; ^4^Istinye University, Department of Radiology, Istanbul, Turkey

## Abstract

**Purpose:**

To search for the utility of DCE-MRP to differentiate between posttreatment enhancement (PT) and tumoral enhancement (TM) in high-grade glial tumors.

**Materials and Methods:**

Thirty-four patients with glioma (11 grade 3; 23 grade 4) were enrolled. Enhancement in the vicinity of the resection cavity demonstrated by DCE-MRP was taken into consideration. Based on the follow-up scans, reoperation or biopsy results, the enhancement type was categorized as PT or TM. Measurements were performed at the enhancing area near the resection cavity (ERC), nearby (NNA) and contralateral nonenhancing areas (CLNA). Perfusion parameters of the ERC were also subtracted from NNA and CLNA. Intragroup comparison (paired sample *t*-test) and intergroup comparison (Student's *t*-test) were made.

**Results:**

There were 7 PTs and 27 TMs. In the PT, the subtracted values of Ve and IAUC from the CLNA and NNA and the subtracted value of Kep from NNA were statistically different. In TM, all metrics were significantly different comparing the CLNA and NNA. Comparing PT with TM, Ktrans, IAUC, Kep, and subtracted values of Ktrans and IAUC from both NNA and CLNA were significantly different.

**Conclusions:**

In PT, only Ktrans values did not reveal any difference comparing NNA and CLNA. To differentiate PT from TM, Ktrans, Kep, IAUC, and subtracted values of Ktrans and IAUC from NNA and CLNA can be used. These findings are in concordance with literature.

## 1. Introduction

High-grade gliomas are aggressive primary brain tumors characterized by high cellularity, anaplasia, mitosis (grade 3), additional microvascular proliferation, and necrosis (grade 4) [1, 2]. CE-MRI is the gold standard noninvasive imaging technique for diagnosis, presurgical planning, and post-therapeutic management of high-grade gliomas. Current best treatment modality consists of maximum safe resection, followed by radiotherapy and chemotherapy. Despite advanced treatment modalities, high-grade gliomas remain almost universally fatal with a median survival of 12–14 months for grade 4 and 3–5 years for grade 3 [3–5]. During the follow-up after operation, control MRI examinations may show either increased/continuing contrast enhancement or new enhancing areas in the resection zone, which may be seen due to posttreatment changes or tumor progression [6, 7]. Radiochemotherapy is the first-line standard treatment applied to patients after resection. Radiotherapy may cause various degrees of vascular permeability changes and blood–brain barrier (BBB) damage [8]. On the other hand, Temozolamide, the first-line chemotherapeutic agent, affects the basal membrane and neovascular endothelium and disrupts permeability. Moreover, postsurgical diffusion restriction at the periphery of the resection cavity in the acute period continues to enhance in the subacute period following 2–3 months after operation. It is not easy to distinguish between posttreatment enhancement (PT) and tumoral enhancement (TM) by conventional contrast-enhanced brain MRI. However, this distinction is essential as it affects follow-up time interval and treatment protocol. Any failure in the evaluation may lead to unnecessary reoperations or premature termination of chemotherapy [8–10].

In the postoperative period, imaging is very limited due to inhomogeneity secondary to blood products and operation material. Postoperative inhomogeneity hinders use of Dynamic Susceptibility Contrast-Enhanced MR perfusion (DSC-MRP) and MR spectroscopy (MRS). Positron emission tomography (PET) and MRS are other advanced imaging techniques used to evaluate treatment efficacy, but their success rates are also limited. Radiation necrosis shows hypometabolism whereas pseudoprogression and true progression shows hypermetabolism on PET scan. Their frequency of use varies according to the clinical experience and technical capabilities of the medical center [10, 11].

Dynamic Contrast Enhanced MR Perfusion (DCE-MRP), a noninvasive advanced MRI technique, has been used lately for tumor grading, tissue segmentation, and to discriminate PT and TM [12]. DCE-MRP has the advantages of being less sensitive to inhomogeneity and the ability of quantification of BBB integrity and the disadvantages of complexity of image acquisition and the lack of widely available easy‐to‐use postprocessing software. On the other hand, lack of standardization in the methodology for parameter computation and lack of cut-off values limit its clinical usage [12]. It is also called as permeability MRI. Tumor or tissue permeability or leakiness is used for data analysis in DCE-MRP, which is considered as an artifact and unwanted situation for DSC-MRP. DCE-MRP is based on two-compartmental pharmacokinetic model (Tofts model), which is produced by the exchange of contrast agent between plasma to the extravascular extracellular space. It provides insights into the nature of tissue properties at microvascular level. According to Tofts model, the perfusion metrics of T1 DCE-MRP include volume transfer constant from the plasma compartment to the extravascular extracellular space (Ktrans), rate constant for transfer from extravascular extracellular space to the blood compartment (Kep), volume of extravascular extracellular space per unit volume of tissue (Ve), volume of the intravascular compartment (Vp), and the initial area under the enhancement curve (IAUC). DCE-MRP metrics provide remarkable details about any specified area [7, 13, 14]. DCE-MRP is becoming more widely available, but standardization in protocols, processing, and postprocessing for uniform interpretation of imaging across institutions is still lacking. In this study, we aimed to search for the utility of DCE-MRP in differentiation of TM and PT on follow-up of patients operated for high-grade gliomas.

## 2. Materials and Methods

### 2.1. Data Collection

Between the dates of December 2015 and March 2019, 34 patients were recruited. Data were retrospectively evaluated. 11 of them were grade 3 glial masses; 23 were grade 4 glial masses. On follow-up, 7 cases showed PT and 27 cases showed TM (Table 1).

All the data were undertaken after total or near total resection for high-grade gliomas. Nearly 10–15 days (wound healing period) after surgery, standard chemoradiotherapy protocols (standard whole brain radiotherapy and temozolamide treatment) were given to all the patients. After completion of radiotherapy, 6 weeks later (nearly 3–3.5 months after the surgery), routine controls of all the patients were performed, including brain MRI, MRP, and MRS. In our institution, postoperative high-grade tumor imaging is routinely performed every 3 months in the first 2 years. Our standard control imaging schemata for the postoperative patients is CE-MRI with DCE-MRP, DSC-MRP, and MRS [15].

Enhancement in the vicinity of the resection cavity (ERC) on DCE-MRP performed at the time of first or second routine control was taken into consideration. None of the patients was treated with gamma knife or antiangiogenic drugs yet. They were followed up postoperatively. If resolved within 6 months after operation, it was called PT. Radiation necrosis and pseudoprogression were all called PT. TM was called when the ERC was getting bigger on the follow-up. Most of the patients underwent biopsy or reoperation and consequently tumor recurrence was proved histopathologically. A few patients were accepted as tumor recurrence based on clinical deterioration and follow-up imaging findings. On tumor progression, gamma knife treatment and/or antiangiogenic drugs were administered.

The study involved a retrospective data review with no risk to the patients. This study was approved by the Institutional Clinical Retrospective Studies Ethical Board (2018.876). All the procedures that were performed involving human participants were in accordance with the ethical standards of the institutional and/or national research committee and with the 1964 Helsinki Declaration and its later amendments or comparable ethical standards.

### 2.2. Chemoradiotherapy Protocol

After 15 days of postoperative wound healing, locally fractionated radiotherapy (60 Gy total dose: 2 Gy × 5 days/week, 6 weeks) with concomitant oral temozolomide (75 mg/m2/day × 7 days/week, 42 days for 6 weeks, maximum 49 days) in the first 10–15 days were given. After that, temozolomide monotherapy (200 mg/m2/day × 5 days, once every 28 days for six cycles) was administered to the patients with newly diagnosed, pathologically confirmed grade 3 and grade 4 glial tumor.

### 2.3. MRI Protocol

MRI was performed on a 1.5 Tesla system (Magnetom Avanto; Siemens Medical Solution, Erlangen, Germany) using a head coil. Conventional contrast-enhanced MRI, DCE-MRP, DSC-MRP, and MRS were performed on routine control of the patients postoperatively. For the postprocessing of DCE-MRP, volumetric anatomic data of the brain is needed. Before intravenous injection of the contrast agent, fast low-angle shot (FLASH) axial 3D T1-weighted images (TR/TE = 6.7/1.0 ms; acquisition matrix = 320 × 384; NEX = 1; field of view = 250 × 300 mm; slice thickness = 5 mm) were acquired with multiple flip angles (5°, 10°, 15°, 20°, and 30°). Acquisition of a DCE-MRI sequence was started immediately after intravenous administration of a gadolinium-based contrast agent (Gadobutrol 0.1 ml/kg, Gadovist) by a power injector (Spectris Solaris EP Medrad) at a rate of 5 mL/s followed by a bolus injection of 15 ml saline. Dynamic axial 3D T1-weighted TurboFLASH images (TR/TE = 6.7/1.0 ms; acquisition matrix = 320 × 384; NEX = 1; FoV = 230 × 300 mm; slice thickness = 5 mm; flip angle = 30°) were acquired for 30 time points. In standard routine imaging, first noncontrast scans of the brain were taken, thereafter DCE-MRP, followed by DSC-MRP, and at last, contrast-enhanced T1W scans and FLAIR images were taken.

### 2.4. Image Analysis

DCE-MRP data postprocessing was conducted by Siemens Syngo via workstation. Pharmacokinetic modeling was performed pixel-by-pixel using a 2-compartment model. Calculation was based on Tofts model. All images and follow-up views were evaluated by a neuroradiologist with 19 years of experience (AA) in a blinded fashion. ERC was chosen after user defined region of interest (ROI) was drawn on the mostly enhancing parts (3‐4 times) in order to find the highest Ktrans value. A nonenhancing area about 1 cm close to ERC was selected as a nearby nonenhancing area (NNA). Another evaluation from contralateral normal appearing, nonenhancing area (CLNA) symmetrical to the ERC was also included. Mean Ktrans, Kep, Ve, and IAUC values were noted at each localization by the same ROI. Furthermore, each parameter measured from ERC was subtracted from the NNA and the CLNA for normalization.

### 2.5. Statistical Analysis

Ktrans, Kep, Ve, and IAUC parameters were measured from ERC, NNA and CLNA. Their values and subtracted values were all noted.

Mean and standard deviation of DCE-MRP metrics measured from ERC, NNA, and CLNA in the PT group are given in Table 2. Intragroup comparison was made by using paired sample *t*-test (Table 3). The same steps were repeated for TM (Tables 4 and 5).

DCE-MRP metrics of ERC, NNA, CLNA, and their subtracted values were compared between the two groups. Intergroup comparison was made by using Student's *t*-test (Table 6). Threshold value for significance was set as *p* < 0.05.

## 3. Results

Between the dates of December 2015 and March 2019, 34 patients were recruited. All were operated for high-grade gliomas. 11 of them were operated for grade 3 glial mass; 23 for grade 4 glial mass. There were 7 PT and 27 TM (Table 1, Figures 1–3).

In TM, compared with NNA and CLNA, Ktrans, Ve, and IAUC were increased while Kep was decreased at ERC. Similar results were found in PT (Tables 2–6).

In Table 2, for the PT group, the mean and standard deviation of DCE-MRP metrics measured from ERC, NNA, and CLNA are given. Comparing the ERC with the CLNA and NNA, Ve and IAUC were found to be statistically different within group evaluation. A statistically significant difference was also found in the Kep values of the ERC compared to the NNA in the PT group. Comparing the CLNA and NNA, Ktrans changes were not found to be significant in PT (Table 3).

In Table 4, for the TM group, the mean and standard deviation of DCE-MRP metrics measured from ERC, NNA, and the CLNA are given. All metrics of DCE-MRP were found to be significantly different in TM compared to the CLNA and NNA (Table 5).

In two-group comparisons, Ktrans, IAUC, Kep, and subtracted values of Ktrans and IUAC from both NNA and CLNA were found to be statistically different. For both of the two groups, mean and standard deviation of DCE-MRP metrics measured from ERC, NNA, and the CLNA, their subtracted values, and intergroup comparison results are given in Table 6.

## 4. Discussion

Treatment options for high-grade gliomas include postoperative radiotherapy and concomitant adjuvant chemotherapy (temozolomide, bevacizumab) [16, 17]. CE-MRI is used to evaluate treatment response [18, 19]. In tumor angiogenesis, poorly formed, anarchic and leaky vessels facilitate an increased uptake of intravenously administered contrast agent in comparison to normal vasculature. Increased vascular permeability forms the basis of TM. Treatment response is assessed by the changes in the contrast-enhancing component of the mass [2, 20]. However, the increase in contrast enhancement after treatment is not always in favor of tumor presence. In the early period, immediately after radiochemotherapy, changes in cell structure and metabolism may result in deterioration of BBB and therefore an increase in contrast enhancement may occur. Stability or reduction of contrast enhancement in size at 6-month follow-up is defined as pseudoprogression or PT [8, 10, 21–23]. Histopathologically, PT is characterized by vascular dilation, fibrinoid necrosis, and endothelial damage of normal cerebral vasculature. Complete PT is higher in patients with O6-methylguanine-methyltransferase (MGMT) promoter methylation and isocitrate dehydrogenase (IDH) mutation [8, 24]. MGMT is known to increase the tumor's sensitivity to the alkylating effects of temozolomide and is associated with increased risk of radiation-induced side effects [24, 25]. High mitotic activity and/or microvascular proliferation in high-grade gliomas make DCE-MRP valuable in the follow-up of suspected areas after treatment. DCE-MRP is a relatively novel imaging modality that combines morphology and hemodynamic changes and can quantitatively evaluate selected tissues [4, 26]. In this retrospective study, we searched for the utility of DCE-MRP metrics in discrimination between the two challenging diagnosis of TM and PT in patients with high-grade gliomas.

The most commonly used DCE-MRP parameter that reflects vascular permeability is Ktrans, which represents the rate at which the contrast agent transfers from the microcirculation to the interstitium. Ktrans gives information about tumor microcirculation and tumoral infiltration. Kep reflects the rate at which the contrast agent transfers from the extravascular extracellular space back to the blood circulation. Ve predominantly reflects the percentage of contrast agent in the extravascular extracellular space (Ve = Ktrans/Kep). Vp reflects fractional volume of the intravascular compartment. IAUC is associated with tumor blood influx and interstitial space and represents the general tumor blood flow, overall perfusion, and tumor interstitial space index [2, 12, 26, 27].

In our study, in TM, when ERC was compared with NNA and CLNA, we found a significant increase in Ktrans, Ve, and IAUC and a decrease in Kep values (Tables 4 and 5). In PT, again an increase in Ve and IAUC and a decrease in Kep values of ERC comparing NNA and CLNA were present (Table 2). The subtracted Ve and IAUC values from both NNA and CLNA and the subtracted Kep values from NNA were found to be significantly different (Table 3). However, subtracted Kep values from CLNA were present but not significant. No significant difference of Ktrans was noted. Ktrans of the ERC was almost similar to that of CLNA and NNA in PT group (Tables 2 and 3).

Distinguishing TM from PT is crucial for treatment management. Misdiagnosis of TM as PT may result in untimely discontinuation of the treatment. On the other hand, incorrect evaluation of PT as TM may lead to improper alteration of the treatment regimen or unnecessary reoperation. PT can sometimes accompany clinical deterioration. This also makes the distinction between TM-PT and treatment management difficult [10, 28, 29].

In our study, when we compared perfusion metrics of the two groups, we found that Ktrans and IAUC values, and their differences from NNA and CLNA were all found significantly different between PT and TM. Kep, on the other hand, was barely different between the two groups (*p* = 0.046) (Table 6). Statistically significant values were as follows: in the ERC, mean Ktrans values of PT vs. TM were 0.01 vs. 0.02 (*p* ≤ 0.001), mean Kep values were 0.52 vs. 0.17 (*p* = 0.046), and the mean IAUC values were 1.58 vs. 2.83 (*p* = 0.016). When the values of ERC were subtracted from CLNA, mean Ktrans values of PT vs. TM were 0.00 vs. 0.02 (*p* = 0,033) and the mean IAUC values were 1.14 vs. 2.42 (*p* = 0.034). When the values of ERC were substracted from NNA and CLNA in both groups, mean Ktrans values of PT vs. TM were 0.00 vs. 0.02 (*p* = 0.001) and the mean IAUC values were 0.69 vs. 1.98 (*p* = 0.012).

Our study is in concordance with the literature. In previous studies, Ktrans and Ve were found valuable for the differentiation between true progression and pseudoprogression [30, 31]. Vp was found to be the most effective metric for distinguishing progression from radiation injury [32]. Zakhari et al. found IAUC and Vp useful in differentiating TM and radiation necrosis [33]. Bisdas et al. found Ktrans and IAUC to be significantly different between tumor recurrence and radiation necrosis and but did not provide Vp results [34]. On the other hand, in a smaller group of patients, Yun et al. found no significant difference in Vp between the two groups [31]. In two different studies, IAUC was found useful in differentiating radiation necrosis from tumor progression in patients with high-grade gliomas [35, 36].

Ktrans denotes permeability and can be affected by endothelial permeability, blood flow, and capillary surface area. Vp has a stronger correlation with the mean vascular area and mean vascular density than Ktrans in glioma [37]. Ktrans can be higher in radiation necrosis due to radiation‐induced endothelial damage. This may be the reason for the lack of Ktrans changes between tumor recurrence and radiation necrosis in some of the previous studies [32, 33]. IAUC describes the initial uptake of contrast agent in a tissue of interest. It has advantages that it does not require arterial input function measurement, is unlikely to be influenced by variations in scanner and sequence type, and does not require complex postprocessing/pharmacokinetic modeling techniques. It includes mixed measurements of tissue blood flow and vascular permeability as well as an indirect measure of the extracellular extravascular space. It is related with blood flow, vessel permeability, and interstitial space. Its physiologic meaning was investigated by Walker-Samuel et al. who showed that IAUC was correlated intractably with Ktrans, extracellular extravascular space volume, and plasma volume [35, 38].

There are limitations of our study. First, we could not measure Vp because of technical reasons. Second, for some of the patients there was no histopathological verifıcation for PT orTM. For some of the patients, our diagnosis of PT or TM was made clinically and imaging based. Third is the absence of subgroups to evaluate the effect of radiotherapy or temozolomide separately in PT. Further studies with these subgroups, with more histopathological verification and with additional measurement of Vp, will provide more useful results in terms of perfusion parameters.

## 5. Conclusion

The distinction between TM and PT in high-grade gliomas is indispensable for the clinician to manage treatment. However, their differentiation in both clinic and imaging wise is still a big challenge. Among the imaging techniques, DCE-MRP looks fascinating since it is noninvasive and less sensitive to inhomogeneity and gives information about tissue permeability and microcirculation but still lacks standardized metrics for interpreting imaging across institutions. In our retrospective study, we found Ktrans, IAUC, Kep, and subtracted values of Ktrans and IAUC from both NNA and CLNA are all valuable in the differentiation of PT and TM in high-grade gliomas.

## Figures and Tables

**Figure 1:** TM is seen at the upper border of the resection cavity in a patient operated for grade 3 glial mass (a). Ktrans, Kep, IAUC maps, and tissue contrast-time curve of DCE-MRP are seen (b). ROIs are placed at ERC, NNA, and CLNA (b). Enhancing area shows the highest permeability with the highest in Ktrans, Ve, and IAUC values and the lowest in Kep values, compared to the other areas.

**Figure 2:** Postcontrast axial T1 (a) and FLAIR images (b) show PT at the ERC in a patient operated for grade 4 glial mass. Ktrans, Ve, IAUC maps, and tissue contrast-time curve of DCE-MRP are seen (c). ROIs are placed at the ERC, NNA, and CLNA(c). Enhancing areas have higher permeability with increased Ve and IAUC but similar Ktrans values compared to the other areas.

**Figure 3:** Postcontrast axial T1 (a) and axial T2 images (b) show PT at ERC in a patient operated for grade 4 glial mass. Ktrans, Kep, IAUC maps, and tissue contrast-time curve of DCE-MRP are seen (c). ROIs are placed at ERC and CLNA. Enhancing areas have higher permeability with increased Ve and IAUC but similar Ktrans values compared to the CLNA.

**Table 1:** The distribution of enhancement type and tumor grade of patients are given in cross-table.

Tumor grade		3	4	Total
Posttreatmeant enhancement	*n*	2	5	7
	%	28.6%	71.4%	100.0%

Tumoral enhancement	*n*	9	18	27
	%	33.3%	66.7%	100.0%

Total	*n*	11	23	34
	%	32.4%	67.6%	100.0%

**Table 2:** Mean and Std deviation of DCE-MRP metrics measured from PT, NNA, and CLNA are given.

T1 DCE MRP metrics	Mean	Std. Deviation
pt ktrans	0.01	0.00
CLNA ktrans	0.01	0.01
pt kep	0.44	0.33
CLNA kep	1.56	1.38
pt ve	0.21	0.13
CLNA ve	0.06	0.05
pt IAUC	1.69	0.39
CLNA IAUC	0.55	0.55
pt ktrans	0.01	0.00
NNA ktrans	0.01	0.01
pt kep	0.44	0.34
NNA kep	1.88	1.52
pt ve	0.23	0.11
NNA ve	0.07	0.06
pt IAUC	1.49	0.45
NNA IAUC	0.80	0.57

**Table 3:** Intragroup comparisons of DCE-MRP metrics measured from PT, NNA, and CLNA are given. Among the permeability metrics of PT, the differences of Ve and IAUC from both NNA and CLNA and the difference of Kep from NNA are significantly different.

T1 DCE MRP metrics	*t*	*p*
pt ktrans – CLNA ktrans	1.581	0.175
pt kep – CLNA kep	−2.093	0.091
pt ve – CLNA ve	2.978	**0.031**
pt IAUC – CLNA IAUC	4.728	**0.005**
pt ktrans – NNA ktrans	−0.542	0.611
pt kep – NNA kep	−2.709	**0.042**
pt ve – NNA ve	5.784	**0.002**
pt IAUC – NNA IAUC	3.059	**0.028**

**Table 4:** Mean and Std deviation of T1 DCE-MRP metrics measured from TM, NNA, and CLNA are given.

T1 DCE MRP metrics	Mean	Std. Deviation
tm ktrans	0.02	0.01
CLNA ktrans	0.01	0.01
tm kep	0.17	0.11
CLNA kep	2.04	1.79
tm ve	0.27	0.15
CLNA ve	0.08	0.08
tm IAUC	2.83	1.30
CLNA IAUC	0.41	0.36
tm ktrans	0.02	0.01
NNA ktrans	0.01	0.01
tm kep	0.14	0.07
NNA kep	1.21	0.75
tm ve	0.28	0.13
NNA ve	0.06	0.08
tm IAUC	2.51	0.97
NNA IAUC	0.53	0.40

**Table 5:** Intragroup comparisons of DCE-MRP metrics measured from TM, NNA, and CLNA are given. Among the permeability metrics of TM, the differences of Ktrans, Kep, Ve, and IAUC from NNA and CLNA are significantly different.

T1 DCE MRP metrics	*t*	*p*
tm ktrans – CLNA ktrans	6.163	**<0.001**
tm kep – CLNA kep	−5.444	**<0.001**
tm ve – CLNA ve	7.364	**<0.001**
tm IAUC – CLNA IAUC	9.030	**<0.001**
tm ktrans – NNA ktrans	6.487	**<0.001**
tm kep – NNA kep	−5.784	**<0.001**
tm ve – NNA ve	5.595	**<0.001**
tm IAUC – NNA IAUC	7.163	**<0.001**

**Table 6:** Mean and Std deviation of DCE-MRP metrics measured from ERC, NNA, and CLNA and their subtracted values are given for both PT and TM groups. Intergroup comparison among permeability metrics, Ktrans, IAUC, and Kep, and the differences of Ktrans and IAUC from both NNA and CLNA are significantly different.

Mean	Std deviation		*t*	*p*	
ERC ktrans	pt	0.01	0.00	−4.291	**0.000**
	tm	0.02	0.01		

ERC kep	pt	0.52	0.37	2.475	**0.046**
	tm	0.17	0.11		

ERC ve	pt	0.20	0.12	−1.075	0.290
	tm	0.27	0.15		

ERC IAUC	pt	1.58	0.47	−2.540	**0.016**
	tm	2.83	1.28		

CLNA ktrans	pt	0.01	0.01	0.332	0.742
	tm	0.01	0.01		

CLNA kep	pt	1.56	1.38	−0.621	0.539
	tm	2.04	1.79		

CLNA ve	pt	0.06	0.05	−0.809	0.425
	tm	0.08	0.08		

CLNA IAUC	pt	0.55	0.55	0.786	0.438
	tm	0.41	0.36		

NNA ktrans	pt	0.01	0.01	1.579	0.131
	tm	0.01	0.01		

NNA kep	pt	1.88	1.52	1.017	0.348
	tm	1.21	0.75		

NNA ve	pt	0.07	0.06	0.163	0.872
	tm	0.06	0.08		

NNA IAUC	pt	0.80	0.57	1.224	0.236
	tm	0.53	0.40		

ERC−CLNA ktrans	pt	0.00	0.01	−2.235	**0.033**
	tm	0.02	0.01		

ERC-CLNA kep	pt	−1.12	1.30	0.987	0.332
	tm	−1.87	1.75		

ERC-CLNA ve	pt	0.15	0.13	−0.547	0.588
	tm	0.19	0.13		

ERC-CLNA IAUC	pt	1.14	0.59	−2.219	**0.034**
	tm	2.42	1.36		

ERC-NNA ktrans	pt	0.00	0.01	−4.019	**0.001**
	tm	0.02	0.01		

ERC-NNA kep	pt	−1.43	1.30	−0.823	0.420
	tm	−1.07	0.72		

ERC-NNA ve	pt	0.16	0.07	−0.898	0.380
	tm	0.22	0.15		

ERC-NNA IAUC	pt	0.69	0.56	−2.772	**0.012**
	tm	1.98	1.07		

## Data Availability

The data used to support the findings of this study are available from the corresponding author upon request.

## Abbreviations

CLNA: Contralateral normal appearing, nonenhancing area
DCE-MRP: Dynamic contrast-enhanced MR perfusion
DSC-MRP: Dynamic susceptibility contrast-enhanced MR perfusion
ERC: Enhancement in the vicinity of the resection cavity
IAUC: Initial area under the enhancement curve
Ktrans: Volume transfer constant from the plasma compartment to the extravascular extracellular space
Kep: Rate constant for transfer from extravascular extracellular space to the blood compartment
NNA: Nearby nonenhancing area
PT: Posttreatment enhancement
PET: Positron emission tomography
ROI: Region of interest
TM: Tumoral enhancement
Ve: Volume of extravascular extracellular space per unit volume of tissue
Vp: Volume of the intravascular compartment.
